This article has been retracted.

# Analysis of Influencing Factors on Hospitalization Expenses of Patients with Breast Malignant Tumor Undergoing Surgery: Based on the Neural Network and Support Vector Machine

**DOI:** 10.1155/2021/9268660

**Published:** 2021-11-24

**Authors:** Jing Zhang, Lin Sun

**Affiliations:** ^1^West China School of Public Health, Sichuan University, Chengdu 610041, Sichuan, China; ^2^West China School of Medicine, Sichuan University, Chengdu 610041, Sichuan, China; ^3^Institute for Hospital Management West China Hospital, Sichuan University, Chengdu 610041, Sichuan, China; ^4^West China Hospital, Sichuan University, Chengdu 610041, Sichuan, China

## Abstract

**Objective:**

Analyze the influencing factors of hospitalization expenses of breast cancer patients in a tertiary hospital in Chengdu and provide a basis and suggestion for controlling the unreasonable increase of medical expenses.

**Methods:**

The first pages of all inpatient medical records of patients with breast malignant tumor from 2017 to 2020 were extracted, and the descriptive analysis, single-factor analysis, and multifactor analysis were conducted by using the statistical method and data mining method to explore the influencing factors of hospitalization expenses.

**Results:**

In 2017–2020, the average hospitalization cost and the average surgical treatment cost increased year by year, and the number of operations, actual hospitalization days, and CCI were the important influencing factors.

**Conclusion:**

It is suggested to strengthen the supervision of medical rationality and eliminate the waste of medical resources; and we should improve the efficiency of diagnosis and treatment services, so as to shorten the actual length of hospitalization; at the same time, the combination of DRG grouping and fine management can be used to control the hospitalization expenses.

## 1. Introduction

In recent years, with the rapid development of social economy, people's demand for health has been increasing, and the problem of waste of health resources is becoming more and more serious in the world. As an important part of medical expenses, hospitalization expenses are paid more and more attention.Slowing down the growth rate of hospitalization costs is the key to solving the problem of overall medical cost growth. At the same time, the treatment of cancer is more likely to incur high medical costs than other diseases. Breast cancer has become one of the most common malignant tumors among women in China [1，^2^]. The annual growth rate of breast cancer-related expenses in China is 2.3%–2.4%, which causes heavy economic burden to individuals and society. How to effectively and reasonably control the growth of medical expenses is of great significance to reduce the disease burden and economic burden of inpatients and society. At present, the management of breast cancer in Chengdu is too extensive, which is not conducive to the reasonable control of hospitalization expenses. Based on the results of this study, the classification of breast cancer in Chengdu area can be further subdivided; at the same time, research idea about this study can be provided for research of other disease, and it also provides theoretical basis and suggestions for improving service efficiency, controlling medical costs, and rationally optimizing medical resources; therefore, it has become an urgent and realistic research topic to explore the important factors that affect the hospitalization expenses of breast cancer patients and to provide a scientific basis for establishing a scientific and reasonable reimbursement mechanism and standard for the hospitalization expenses of breast cancer patients.

## 2. Information and Methods

1. Source of information: the data of this study came from the medical record information management system of a general third-class hospital in Chengdu. In order to ensure the integrity and systematicness of the data,the relevant data information on the first page of medical records of all discharged patients diagnosed with breast malignant tumors in the hospital from January 1, 2017, to December 31, 2020, were derived from the system, and then the patients undergoing breast malignant tumor surgery were selected according to the diagnostic code and operation code. Finally, the selected data were used to establish the initial patient database. The patients with malignant breast tumor were selected, and the initial patient database was established. Finally, the repeat cases, main information missing cases, and the abnormal cases whose hospitalization days <1 or >60 were eliminatedor the total hospitalization cost was beyond P1–P99.
2. Method: Excel was used to analyze the composition ratio and development trend of hospitalization expenses, and then a single-factor analysis was performed to determine the relationship between different demographic characteristics, disease characteristics, and total hospital costs for breast cancer patients. Based on the results of the normality test and related literature, the total cost of hospitalization and the single cost all present a skewness distribution. Therefore, nonparametric test was used to analyze the cost of hospitalization under each influencing factor. In the non-parametric test, Mann–Whitney *U* test was used for two independent samples, and Kruskal–Wallis *H* test was used for many independent samples. The test level *α* = 0.05 was used to screen out the influential factors which had statistical significance on hospitalization expenses ,finally multi-factor analysis was used to further analyze the degree of influence of each factor on hospitalization expenses, and then the important influencing factors are explored.” Regression analysis has been widely used in the previous analysis of influencing factors, but many studies using regression analysis have not reported in the paper whether it meets the preconditions of regression analysis: normality, independence, linearity, variance equality, etc. hospitalization cost is a kind of medical big data. Compared with the general data, the information of hospitalization cost has the characteristics of skewness and correlation among variables. Therefore, the traditional regression analysis method often has the limitation in the study of hospitalization cost and is no longer sufficient for analysis. Some research studies show that the fitting result of the data mining method may be more suitable for medical big data [3], such as artificial neural network (ANN) and support vector machine (SVM) [4]. This study used the above two methods to carry out the multifactor analysis on the influencing factors of the hospitalization expense, compared the forecast performance of the two results, and chose the suitable model as the final result. In the above factor analysis, CC method was used to analyze the coincidence and complications quantitatively [5], and the CCI of each case was calculated as a new variable in the factor analysis.

## 3. Results

1. Descriptive statistics of hospital expenses: the results, as shown in Table 1 and Figure 1, were 33% for diagnosis and 31% for surgery, and the rates of medical materials, drugs, nonoperative treatment, and service were 11%, 8%, 7%, and 3%, respectively. The trend of the average cost was evaluated by the line graph drawn by Excel, and the results are shown in Figure 2: in 2017–2020, the average cost was 21239.01489RMB, 22057.25477RMB, 23050.40358RMB, and 23048.36969RMB, respectively. The cost of operation was 29.56%, 29.67%, 31.20%, and 32.60%, respectively. The cost of diagnosis was 34.97%, 35.18%, 33.73%, and 30.80%, respectively. And the cost of medical materials was 11.09%, 11.15%, 08.30%, and 12.49%, respectively.
2. Calculation of CCI (score of complications): the following steps are included: (1) calculate the frequency of each complication, and combine the complications with frequency less than 5 into others; (2) establish the complication table of patients: count the complications of each patient; (3) calculate the weight coefficient of complications: take the total cost after logarithmic conversion as the dependent variable and the presence or absence of complications (0/1) of patients as the independent variable to establish a multiple linear regression model. The regression coefficient in the model output result is the weight coefficient of complications, indicating the impact of this CC category on medical resources. If the coefficient is negative or *P* ≥ 0.05, it means that the CC category has no impact on the consumption of medical resources, and its weight value is treated as 0; (4) calculate the patient's complication score CCI: the sum of the corresponding weight coefficients of the complications of the case. The results are shown in Tables 2 and 3.
3. Single-factor analysis of hospitalization expenses: because the cost of hospitalization does not satisfy the conditions of the parameter test, we used nonparameter test to analyze the cost of hospitalization under each influencing factor, and Kruskal–Wallis test was used to test the data from multiple independent samples. The test level was α = 0.05. The influencing factors of hospitalization expenses were analyzed. The results are shown in Table 4. The influencing factors that have statistical significance on hospitalization expenses are age, mode of payment, length of stay, number of operations, operative grade, and CCI.
4. Multifactor analysis of hospitalization expenses: artificial neural network can be regarded as a computer-intensive classification method. Theoretically, artificial neural networks should have considerable advantages over standard statistical methods, such as allowing double nonlinear relationships between independent variables and dependent variables and all possible interactions between dependent variables [6]. Support vector machine is a new general learning method developed on the basis of statistical learning theory. Based on the VC dimension theory of statistical learning theory and the principle of structural risk minimization, it seeks the best compromise between the complexity of the model and learning ability according to the limited sample information, so as to obtain the best generalization ability [7]. In this study, the neural network and support vector machine were used simultaneously to explore the factors that had the greatest impact on hospital costs. According to the results of univariate analysis, the input variables included age, mode of payment, length of stay, number of operations, operative grade, and CCI. Using SPSS Modeler software to build the model and using the indexes of error and correlation coefficient, the model with good fitting effect was selected as the result of multifactor analysis. The results are shown in Table 5. In each evaluation index, the average absolute error represents the proximity between the predicted value and the real value. The smaller the value, the higher the prediction accuracy of the model. The correlation coefficient is the index to evaluate the goodness of fit of the model. The larger the value, the better the model fitting. The correlation coefficient and error showed that the fitting effect of the neural network model is better than that of the support vector machine. Therefore, the output of the neural network model was selected as the final result of the multifactor analysis, as shown in Table 6. As you can see from the neural network output, the order of importance of the factors influencing the hospitalization expenses of patients with breast malignant tumor was the number of operations (0.49), the actual length of stay (0.35), the CCI (0.14), the age (0.03), the level of operation (0.03), and the mode of payment (0.01).

## 4. Conclusion

1. The general situation of hospitalization expenses of patients with breast malignant tumor operation: the highest proportion of hospitalization expenses is diagnosis expenses, which is 33%, followed by operation treatment expenses and medical material expenses, which are 31% and 11%, respectively; the remaining service fees, drug fees, nonsurgical treatment fees, and other fees account for a relatively low proportion. The operation fees and diagnostic fees account for a large proportion of the cost of cancer in line with the current structure of the common situation in China. In the trend chart, the average total cost and the large proportion of the average cost of surgical treatment increased year by year, while the average cost of medical materials decreased significantly in 2019; the reason may be related to the management upgrade of medical consumables in the 2019 medical reform and the cancellation of the consumable bonus in public hospitals [8].
2. According to the results of neural network analysis, the most important influencing factor is the number of operations, and there is a positive correlation between the number of operations and the cost of hospitalization. The more the operations, the higher the cost of hospitalization, for the surgical treatment of malignant tumors, the more complicated the disease is, and the more surgery is often needed at the same time or successively in order to achieve the desired therapeutic effect; multiple operations represent high operating and hospitalization costs and should also pay attention to whether there are unreasonable treatment and waste of medical resources. Therefore, the number of operations is an important influencing factor for hospitalization costs. When grouping related diseases, the number of operations should also be taken into account, so as to make fine segmentation. Secondly Less important was the actual length of stay, which showed that the longer the stay, the higher the cost. The reasons for this situation have their rationality and irrationality. For example, it is normal for difficult cases to have relatively long hospitalization days and relatively high hospitalization expenses, but it is not reasonable if the hospitalization time is deliberately prolonged; therefore, it is suggested that reducing the average length of stay is an effective way to control the cost of hospitalization on the premise of achieving the goal of treatment and ensuring the efficiency of treatment. Thirdly, there is a positive correlation between the CCI and the cost of hospitalization. The higher the CCI is, the more the complications are; therefore, the cost of operations such as the number of operations discussed above, the cost of diagnosis, and the cost of materials will increase accordingly, so CCI is a noteworthy influencing factor. The effect of age, grade of operation, and payment method is relatively small; that is, the older the age, the higher the cost of hospitalization; the reason may be that the health status declines with age, and the consumption of medical resources increases. In addition, the medical expense of urban workers is higher than that of urban and rural residents, and the difference has statistical significance. It is speculated that it may be related to the higher proportion of medical insurance reimbursement of urban workers, which, to some extent, reflects the waste of medical resources and deserves attention and adjustment.

To sum up, based on the results of this study, the number of operations, length of stay, and CCI are the most important influencing factors. Combining the analysis of the above factors, some suggestions are made to control the increase of hospitalization expenses. First, strengthen the supervision of medical rationality, and put an end to the malicious increase of unnecessary treatment and waste of medical resources. Second, improve the efficiency of diagnosis and treatment service, strengthen the innovation of the service process, and prevent unreasonable extension of hospital stay, thus shortening the actual length of hospital stay, and control hospital costs. Third, according to the important factors and the opportunity of DRG development, the cases can be divided into small groups, so as to carry out standardized management and improve management efficiency.

## Figures and Tables

**Figure 1:** Chart of inpatient costs for breast cancer surgery.

**Figure 2:** Trend of average cost per hospitalization in patients undergoing breast cancer surgery.

**Table 1:** Composition of hospitalization expenses of patients with breast malignant tumor undergoing surgery.

	Service charge	Diagnostic fee	Nursing expenses	Surgical expenses	Nonsurgical expenses	Medical expenses	Cost of blood products	Cost of medical materials	Other expenses
Total cost	2143819	23236847.69	846926.18	21657109.73	4931820.27	5364841.26	66712.65	7292302.98	4119887.88
Percentage	3.077534831	33.35739077	1.215795185	31.08961602	7.079818148	7.701436474	0.095768581	10.46838209	5.914257897

**Table 2:** Weight coefficient of complications in patients undergoing breast cancer surgery.

Variable (code for complications)	Coefficient	*t*	Statistical significance
Constant		1201.422	0.000
C77.301	0.102	5.904	0.000
N39.000	0.116	6.810	0.000
D24.x00	0.101	5.614	0.000
Z51.103	0.104	6.123	0.000
J94.804	0.082	4.813	0.000
E77.801	0.070	4.077	0.000
N60.201	0.076	4.216	0.000
C50.100	0.061	3.657	0.000
R94.303	−0.052	−3.080	0.002
In the news	0.062	3.600	0.000
K76.000X011	−0.054	−3.177	0.002
J34.300	0.066	3.611	0.000
Z85.300	−0.048	−2.836	0.005
M50.201	−0.055	−3.240	0.001
N63.x00	0.054	3.122	0.002
D61.101	0.051	2.994	0.003
D05.100x001	0.048	2.839	0.005
C79.800X809	0.059	3.349	0.001
N64.802	0.045	2.672	0.008
N64.500	0.045	2.671	0.008
D69.600	−0.043	−2.575	0.010
T85.400	0.044	2.585	0.010
D48.601	0.042	2.503	0.012
J34.200	−0.041	−2.280	0.023
I 82.804	0.042	2.481	0.013
N63.X01	0.040	2.290	0.022
C50.300	0.039	2.296	0.022
R90.000x002	0.037	2.211	0.027
J47.x00	−0.035	−2.062	0.039
J47.x03	−0.036	−2.134	0.033
C50.200	0.036	2.157	0.031
D72.800x002	0.036	2.136	0.033
C77.002	0.036	2.111	0.035
C50.800	0.035	2.072	0.038
F41.101	0.034	2.024	0.043
R22.201	0.038	2.226	0.026
C79.827	−0.044	−2.456	0.014
M48.901	0.038	2.209	0.027
N64.503	0.034	1.994	0.046

**Table 3:** CCI of breast cancer surgery patients in a hospital in Chengdu from 2017 to 2020.

Period	ID code	CCI
202010	00001	0.376190627
202012	00002	0.361690004
201911	00003	0.360015743
202001	00004	0.360015743
201807	00005	0.336938059
202004	00006	0.333024001
202010	00007	0.332539654
201801	00008	0.332539654
201906	00009	0.332539654
201803	00010	0.332539654
201807	00011	0.332539654
201908	00012	0.332539654
201904	00013	0.332539654
201904	00014	0.332539654
202012	00015	0.332539654
201812	00016	0.329251529
202004	00017	0.317962384
202009	00018	0.317962384
201911	00019	0.317962384

**Table 4:** Results of univariate analysis.

Variable	Mean value	Number of cases	Standard deviation	Median	Percentage	*P*
Age						<0.01
≤20	32690.335	2	19054.86605	32690.335	0.10%	
20–40	25901.0894	510	11065.29952	22159.69	1660	
40–60	21960.9184	1999	8141.2137	20451.57	65.10%	
60–80	21875.2406	549	8520.29518	20260.46	1790	
>80	43268.0291	11	69149.33435	23239.59	0.40%	

Native place						0.143
Unknown	19341.674	5	2741.14545	19720.7	0.20%	
Southwest	22658.015	2878	9858.99858	20671.02	93.70%	
Northwest	23791.9147	58	8828.24487	21380.105	1.90%	
East China	23717.2767	43	10817.21822	21175.99	1.40%	
Central China	22486.9883	35	6097.92305	21411.29	1.10%	
North China	24536.2174	23	9262.9743	21481.48	0.70%	
Northeast	21610.6044	18	9009.82898	18054.66	0.60%	
South China	19422.6918	11	5458.59496	18884.54	0.40%	

Nation						0.324
Han nationality	22771.8336	2755	10061.9057	20701.26	89.70%	
Tibetan	21321.5037	54	5155.2445	20224.15	1.80%	
Others	22032.4616	262	7269.37178	20308.155	8.50%	

Occupation						0.204
Farmers	21743.1218	393	8285.32421	20478	1280	
Staff	23347.5746	276	8349.4663	20900.1	9.00%	
Technical expertise	23687.8992	194	10295.17455	20883.69	6.30%	
Retiree	21977.3684	187	7338.63312	20163.83	6.10%	
Civil servants	23720.3678	129	10649.82274	20764.4	4.20%	
Others	22677.6651	1892	10342.75743	20684.605	61.60%	

Payment method						<0.01
Others	22426.4669	2019	10437.36182	20472.57	65.70%	
Town employee	23297.1823	890	8726.14502	20970.715	29.00%	
Urban and rural residents	22510.7327	162	6230.07858	21368.69	5.30%	

Length of stay						<0.01
≤5	19413.8759	192	9231.37935	18080.63	6.30%	
5–10	22163.7347	2711	7072.05057	20566	88.30%	
10–15	29557.7026	139	11623.11149	26396.88	4.50%	
>15	59944.759	29	51470.89992	44091.36	0.90%	

Mode of discharge						0.835
Doctor's orders	22682.5627	3060	9800.73906	20681.395	99.60%	
Transfer on doctor's orders	23104.706	10	6806.35353	23218.545	0.30%	
Death	20578.81	1	.	20578.81	0.00%	

Pathological diagnosis						0.173
Not subdivided	22393.1364	2062	7561.24753	20752.235	67.10%	
Noninvasive	21711.0832	37	12369.74946	19623.81	1.20%	
Invasive special carcinoma	21745.2973	48	8192.17301	20354.835	1.60%	
Invasive nonspecific carcinoma	23464.1058	901	13552.86947	20595.15	29.30%	
Others	21625.0744	23	8582.79677	19170.54	0.70%	

Number of operations						<0.01
≤2	20105.6137	1311	5798.30993	19396.58	42.70%	
3–5	23171.5636	1422	7833.40981	21445.445	46.30%	
>5	30626.7595	338	19838.96913	26006.47	11.00%	

Surgical grade						<0.01
Level 1	26477.6325	4	9519.5442	23846.445	0.10%	
Level 2	22797.0614	7	6439.33718	21836.76	0.20%	
Level 3	20577.9487	780	5128.11815	20074.74	25.40%	
Level 4	23396.4814	2280	10855.72205	20950.575	74.20%	

Readmission status						0.3
Yes	24688.615	453	17439.8389	20919.71	1480	
No	22322.3023	2614	7655.06889	20633.945	85.10%	
Unknown	31456.6875	4	19889.14619	21774.065	0.10%	

CCI						<0.01
0	20700.5261	1013	5843.80473	19872.92	33.00%	
0–0.1	22070.1947	729	8176.88359	20012.11	23.70%	
0.1–0.2	23492.7826	1160	8921.19155	21512.5	37.80%	
0.2–0.3	31261.7223	146	22471.80424	25929.435	4.80%	
0.3–0.4	34157.5413	23	34880.01899	25107.19	0.70%	

Rh						0.07088
Unknown	22014.4542	704	7794.55932	20411.13	0.229	
Positive	22882.3501	2347	10329.55077	20750.74	0.764	
Negative	22860.81	20	6557.75538	21618.945	0.007	

Allergies						0.005164
Yes	22210.7861	1568	6655.0434	20969.485	0.511	
No	23176.151	1503	12215.7928	20278.69	0.489	

**Table 5:** Comparison of neural network and support vector machine fitting.

	Support vector machine		Neural network	
	Training set	Test set	Training set	Test set
Minimum error	−0.95	−0.894	−0.22	−0.505
Maximum error	1.064	0.892	0.221	0.528
Mean error	−0.007	−0.006	−0.006	−0.004
Mean absolute error	0.213	0.217	0.067	0.081
Standard deviation	0.274	0.273	0.084	0.113
Correlation	0.331	0.263	0.741	0.474
Occurrence rate	2,422	649	2,422	649

**Table 6:** Importance ranking of neural network variables.

Nodes	Importance
The mode of payment	0.0024
Age	0.0334
Level of operation	0.034
CCI	0.1428
Actual length of stay	0.3533
Number of operations	0.4341

## Data Availability

No data were used to support this study.
